The article "A Cumulants-Based Human Brain Decoding" was published in 2022. Journal: Comput Intell Neurosci.

# A Cumulants-Based Human Brain Decoding

**DOI:** 10.1155/2022/6474515

**Published:** 2022-07-11

**Authors:** Raheel Zafar, Muhammad Javvad ur Rehman, Sheraz Alam, Muhammad Arslan Khan, Asad Hussain, Rana Fayyaz Ahmad, Faruque Reza, Rifat Jahan

**Affiliations:** ^1^Faculty of Engineering and Computer Science, National University of Modern Languages, Islamabad, Pakistan; ^2^Department of Computer Science & Engineering, HITEC University, Museum Road, Taxila, Pakistan; ^3^Centre for Intelligent Signal and Imaging Research, Universiti Teknologi PETRONAS, Seri Iskandar 32610, Perak, Malaysia; ^4^Center for Neuroscience Services and Research, Universiti Sains Malaysia, Kubang Kerian 16150, Kota Bharu, Kelantan, Malaysia; ^5^Department of Electronics and Telecommunication Engineering, Rajshahi University of Engineering & Technology (RUET), Rajshahi 6204, Bangladesh

## Abstract

Human cognition is influenced by the way the nervous system processes information and is linked to this mechanical explanation of the human body's cognitive function. Accuracy is the key emphasis in neuroscience which may be enhanced by utilising new hardware, mathematical, statistical, and computational methodologies. Feature extraction and feature selection also play a crucial function in gaining improved accuracy since the proper characteristics can identify brain states efficiently. However, both feature extraction and selection procedures are dependent on mathematical and statistical techniques which implies that mathematical and statistical techniques have a direct or indirect influence on prediction accuracy. The forthcoming challenges of the brain-computer interface necessitate a thorough critical understanding of the complicated structure and uncertain behavior of the brain. It is impossible to upgrade hardware periodically, and thus, an option is necessary to collect maximum information from the brain against varied actions. The mathematical and statistical combination could be the ideal answer for neuroscientists which can be utilised for feature extraction, feature selection, and classification. That is why in this research a statistical technique is offered together with specialised feature extraction and selection methods to increase the accuracy. A score fusion function is changed utilising an enhanced cumulants-driven likelihood ratio test employing multivariate pattern analysis. Functional MRI data were acquired from 12 patients versus a visual test that comprises of pictures from five distinct categories. After cleaning the data, feature extraction and selection were done using mathematical approaches, and lastly, the best match of the projected class was established using the likelihood ratio test. To validate the suggested approach, it is compared with the current methods reported in recent research.

The article "A Cumulants-Based Human Brain Decoding" was published in 2022. Journal: Comput Intell Neurosci.

## 1. Introduction

The significance of neuroscience has become iconic in recent years due to the demand for intelligent systems in daily life. In the last decade, neuroscience becomes very famous due to its tremendous advances and applications. Neuroscientists from all over the world have progressed in this area; individual investigators also played a vital role in this field and worked in small groups on specific projects. Since neuroscience is an emerging field and has enormous applications, and therefore, during the last decade, a huge amount of funding is provided. In 2013, US President approved a grant of USD 100 million to unlock the mysteries of the brain [1]. Similarly, in 2013, the European Union [2] also approved funding of 1 billion Euros for human brain projects. The main driving force in the field is the impact of brain disease on the population and the knowledge gaps in neuroscience, requiring a collaborative large-scale effort of scientists. The increasing demand for this field is due to its strength as it can be used in various fields. From medical to defense, it can be used in any field including trials in court and as a basic research tool. Previously, it was used as evidence by the court in India [3], also used in various medical applications [4], and can be used for defense purposes [5, 6]. It can also be used to see the effect of the brain on various products. A blind test was done between Pepsi and Coke based on functional magnetic resonance imaging (fMRI) data to see which one is better [7]. The results showed that although Coke is a more valuable and successful brand, more people liked Pepsi. In Baylor College of Medicine, Houston performed another research in which fMRI data were used to see the brain activations for the taste of Pepsi and Coke [8]. The participants drank Pepsi or Coke and different parts of the brain light up depending on the cola being drunk. A linear regression analysis using behavioral preferences indicated the difference in brain responses evoked by Coke and Pepsi in the ventromedial prefrontal cortex. The average count was higher for labeled Coke compared to the labeled Pepsi. This shows that high activation was found when the participant drank their favorite cola. It is concluded that if acceptable accuracy can be achieved, then the prediction of the human brain can help in many applications including medical and health care.

In the above paragraph, the importance of prediction is discussed that how it can change our lives. Although several other applications are dependent on this field [9–11], the purpose of this paper is not to mention all the applications as they will be beyond the scope. The primary question that arises in the current situation is why we are not using this field for various applications as discussed above, for example, in court trials, and it is easy to predict from a suspect's brain measure whether he/she is involved in crime or not. The answer is it is not possible till now due to limited accuracy and reliability.

The article "A Cumulants-Based Human Brain Decoding" was published in 2022. Journal: Comput Intell Neurosci.

This research work comes under the field of computational neuroscience which uses theoretical neuroscience to validate and crack computational models. This should also be seen as a domain of theoretical neuroscience, but both areas are mostly related. The word mathematical neuroscience is used to emphasize the numerical character of the discipline occasionally [12, 13]. Computational neuroscience focuses on the description and physiology of biologically plausible neurons (and neural systems) as well as their dynamics, but biologically unreal models used for relativism, theory of control, cybernetics, quantitative psychology, machine learning, artificial neural networks, artificial intelligence, and computer education are not directly involved [14, 15]. While there is shared motivation and often no strict boundary within disciplines, paradigm abstractions depend on the complexity of the study and on the functionality by which biological structures are evaluated in computational neuroscience. In the current study, a method is proposed that can improve the accuracy and hence make this field more reliable. There are different steps from experiment design to the prediction of the class including data collection, feature extraction, and selection as shown in Figure 1. Different studies focused on different steps, but the common goal was to achieve better accuracy [16, 17]. For example, a better experiment design can improve prediction accuracy, and similarly, by collecting quality data, accuracy can be improved. In short, the current research is mainly focusing on the analysis of fMRI data instead of depending on new hardware so in this study we have also focused to improve the accuracy by introducing a novel method. Since fMRI is a mature modality in neuroscience and is used for two decades, a lot of literature is available, and various techniques are used for better results. The primary focus of these studies was on experiment design and specific brain regions instead of new statistical techniques like many studies that used a support vector machine (SVM) for classification and took features from the region of interest (ROI) [17–20]. Therefore, the target of this study is to introduce a novel method in neuroscience and compare the results with the existing methods.

The article "A Cumulants-Based Human Brain Decoding" was published in 2022. Journal: Comput Intell Neurosci.

Prediction of the human brain is always a challenging task for neuroscientists due to its complex structure and rapid changing behavior. In the initial years of research, univariate-based approaches were very common and provided acceptable results [21, 22]. Univariate is the simplest form of analyzing data in which the data being analyzed contains only one variable. As univariate has a single variable, it does not deal with relationships or causes. Over time, improvements were done not only in hardware but new methods were also introduced for the analysis of complex brain data. Instead of univariate analysis, brain mapping and multivariate pattern analysis (MVPA) were introduced which improved the previous results significantly [17, 23, 24]. In MVPA, the primary focus is on distributed patterns of activity for analysis and comparison. In this way, the differences between different brain conditions can be detected with higher sensitivity.

In the initial years, functional magnetic resonance imaging (fMRI) was the most common, reliable, and widely used approach for the collection of brain data [22, 25], and in most of the initial studies, the data were extracted only from a particular brain region like occipital region for any visual task or from a temporal region in case of a cognitive task. As time passes, other modalities were also extensively used in neuroscience which provided good results such as an electroencephalogram (EEG), magnetoencephalography (MEG), and functional near-infrared spectroscopy (fNIRS) [26, 27]. In fMRI, brain activity is measured by identifying the changes that occurred due to the flow of blood. The fMRI uses the blood oxygen level-dependent (BOLD) contrast which was initially discovered by Seiji Ogawa [28]. In case of any neuronal activity, more blood is needed in that region which later flows and increases the blood level in that region. Due to blood flow, more BOLD contrast can be observed in that region. Since, in fMRI, brain activity is measured using blood flow, it is an indirect method to measure brain activity. Functional MRI is an indirect method of measuring brain activity patterns, but still the best among other modalities due to its higher spatial resolution. On the other hand, in EEG, the direct neuronal activity can be measured as its time resolution is in milliseconds, which is good compared to fMRI as it has in seconds.

The collection of brain data is itself a difficult task including experiment design and conduction. However, after the recording of brain data, the primary goal is to clean the data and find a significant difference in the temporal and spatial characteristics of the data, which contrasts the various states as precisely as possible. The goal of neuro-computing is to achieve this precise contrast, so a variety of simple and traditional statistical methods such as grand averages and region of interest were used in building the good model [22, 29, 30]. Currently, these methods are not common due to limited accuracy and reliability in comparison with new and complex statistical methods [20, 31, 32]. Although it is not possible to measure and analyze the billions of neurons present in the brain and none of the current modalities can do that, improvement is always demanding and challenging. Moreover, it is not easy to update the hardware regularly. That is why presently the focus of neuroscientists is on computations based on statistical and machine learning techniques which are applied in various fields, to improve the results instead of waiting for new technology [33–36].

The article "A Cumulants-Based Human Brain Decoding" was published in 2022. Journal: Comput Intell Neurosci.

Various research groups are working on neuro-computing, and improvements have already been observed both in terms of hardware and computational techniques, but this field still has a lot of potentials. Neuroscientists also used both fMRI and EEG together (simultaneously) in some studies [37–39] for improved results. In short, this field still has a chance of improvement in many ways. In hardware improvements, 7 Tesla fMRI machines and 512 channel EEG caps are available, and researchers are focusing on statistical and mathematical approaches to bring advancement in existing techniques with the help of advanced hardware. Many novel approaches are observed during the last decade, especially for feature extraction, feature selection, and prediction [26, 40]. Various projection and dimension reduction methods also emerged for the extraction of significant data. The common algorithms used for feature extraction are principal component analysis (PCA), independent component analysis (ICA), *t*-test, and many others [17, 41–43].

Apart from the above-discussed techniques, machine learning plays a vital role in the prediction of brain activities as the brain consists of a huge amount of data. Different machine learning and prediction techniques are used in this regard such as linear discriminant analysis (LDA), support vector machines (SVM), Naïve Bayes, Bayesian, and many others [42, 44–51]. Each of them took part in better results; however, SVM is the most common in neuroscience compared to others. The likelihood ratio test (LRT) is also a statistical test used for comparing the best fit of two statistical models. LRT has mostly been used in likelihood ratio-based score fusion (LRBSF) which is a mature and widely used technique, especially in biometric systems [52], and however, it is rarely used in the neuroscience research area. In an existing study, [53], it was shown that LRBSF can produce better results in terms of accuracy for both fMRI and EEG data sets as compared to many existing methods, especially SVM.

The article "A Cumulants-Based Human Brain Decoding" was published in 2022. Journal: Comput Intell Neurosci.

### 1.1. Contribution of the Research

In this manuscript, a hybrid method is proposed. In the proposed algorithm, time series mathematical equations of various cumulants are used along with the likelihood ratio-based score fusion (LRBSF) method. The results are compared with the recent state-of-the-art methods. In the proposed method, the initial *β* values are taken as features that are found using GLM. These features are further refined with various orders (up to fourth) of cumulants and finally used likelihood ratio-based score fusion (LRBSF) which helped in better results with less time. In LRBSF, the number of features plays a great role, and limited features increase the performance by reducing the processing time of the existing method other than the prediction results.

### 1.2. Organization of the Article

The rest of the paper is organized as follows.  Section 2 presents the experimental methodology of this paper.  Section 3 deals with the statistical techniques which are mainly used in this research article.  Section 4 represents the results based on the experimental setup, and a detailed discussion is given in the section. In the last Section 5, a conclusion of this research work is presented.

## 2. Experimental Methodology

The motivation behind the presented research work is to propose a method based on cumulants that can help in improving the accuracy using the fMRI data because the implementation of neuroscience applications is dependent on higher accuracy. The reliability of any method is dependent on accuracy; if the accuracy is higher, the method is considered accurate and reliable. Cumulants are widely adopted in classification problems such as modulation recognition [54, 55]. To the best of our knowledge, this approach is seldom explored for fMRI analysis. Therefore, a novel prediction approach of cumulants-driven likelihood ratio-based score fusion (LRBSF) along with multivariate pattern analysis (MVPA) is presented in this research article to optimize the prediction results based on the fMRI data set.

For this study, the experiment was designed in e-prime [56], and fMRI was collected using a 3 T Philips machine and preprocessed using standard preprocessing methods in SPM [57]. During analysis, raw data were taken as features that were followed by feature selection done using a *t*-test. Multivariate pattern analysis (MVPA) has been used with fMRI data to extract information from distributed activation patterns of the brain. The significant features were still in large numbers, so different orders of cumulants were applied to reduce the number of features. Finally, the likelihood ratio test (LRT) was applied to those selected features and found the prediction accuracy.

The article "A Cumulants-Based Human Brain Decoding" was published in 2022. Journal: Comput Intell Neurosci.

The main steps of fMRI data analysis include experiment design, data collection, preprocessing, data transformation, data selection, feature extraction, prediction, and finally, results which are shown in Figure 1, and details are given in the following section.

### 2.1. Experiment Design

The initial step is the experiment design which helps in the extraction of data from the brain. Better experiment design can collect valuable and numerous data from the brain like event-related design, which helps in measuring the rapid change of brain-behavior. For the fMRI study, experiment design is an important factor as fMRI scans are expensive and time-consuming and need human resources. That is why experiment design should be carefully designed which can extract sufficient data for further analysis. The best experiment design can maximize the contrast of interest.

### 2.2. Experimental Data Collection

After the experiment design, data collection is a key step in which extensive care is required to retrieve useful data. The main goal during data collection is to record the data according to the task with the minimum artifacts or noise. In fMRI, data collection requires special consideration. The collected data should have strong physiological signals so that the discrimination between the brain states can be done easily along with the safety measures due to human involvement. For the experimental setup, healthy subjects were selected, and all were Hospital Universiti Sains Malaysia (HUSM) students. Their ages were between 18 and 26. The approval of the study protocol was taken from the Human Research Ethics Committee (HREC), Universiti Sains Malaysia (USM) under IRB Reg. No: 00004494, FWA Reg. No: 00007718, and USM issuing letter number is USMKK/PPP/JEPeM[257.3.(4)]. Therefore, it does not require registration with the International Committee of Medical Journal Editors (ICMJE). The consent from all participants (subjects) was obtained before the start of the experiment. For safety purposes, the data were recorded in the company of the doctor at HUSM. A brief training session was arranged for each participant before the data collection.

Subject selection and machine parameters should precisely be chosen. Moreover, the duration of the session should not be too long. In this study, the data were collected from 12 subjects, and 8 were used for the analysis as data of 4 subjects were excluded due to artifacts and low accuracy. A total of 260 images were shown to the subjects in three different sessions, and all the images were grayscale images. These images were taken from the study [53] and are available online. These images were belonging to five different categories as described earlier means a picture of a human or animal or fruit or natural scene or building was presented to the subject. The subject should see the image carefully and recognize the category or class of the image. The target of the study is to see and find the differences in brain activities for various types of images significantly, in other words, to know whether the brain behaves differently for different categories.

The article "A Cumulants-Based Human Brain Decoding" was published in 2022. Journal: Comput Intell Neurosci.

Functional MRI data were collected using 3 Tesla machines with response time (TR)=2000 ms, echo time (TE)=30 ms. After every 2 second, 35 slices of the brain were taken. The anatomical data of 5 mins were separately taken which was later used during the registration of functional images with a structural MRI image. The preprocessing of the data was done using SPM 8. All the gradient echo-planar imaging (EPI) images were realigned to the first image as it has minimum head movement. The normalization was done using the Montreal Neurological Institute (MNI) space, and spatial smoothing was done with a voxel size of 3 × 3 × 3 mm. The final dimension of each fMRI image is 63 × 53 × 46. The proposed method is trained and tested along with other methods that are used as the baseline compared to the proposed method. The reported results are with 8 subjects, and the average accuracy of them is mentioned in the result section.

### 2.3. Preprocessing

Preprocessing also plays a vital role during the analysis as it detects and reduces most of the artifacts and noise from the data. The main steps involved in preprocessing are slice timing correction, realignment, coregistration, segmentation, spatial normalization, and smoothing. In slice time correction, the differences in slice acquisition times are corrected. This correction is required to make the data on each slice correspond to the same point in time. The realignment process detects and corrects the motion of the subject inside the scanner during recording. During the process of coregistration, the functional images (T2) are aligned with the anatomical MRI images also known as T1 or structural images. In segmentation, the gray matter, white matter, and cerebral spinal fluid are separated and can be seen separately. Since every brain size is different, normalization is done to put the different scanned images into a standard Montreal Neurological Institute (MNI) template. The standard MNI template is based on the average of MRI scans of healthy subjects. In smoothing, average values of the neighbor voxels are found for minimal noise. This is the last step of preprocessing which blurs the fMRI image by giving different weights based on the Gaussian kernel.

The article "A Cumulants-Based Human Brain Decoding" was published in 2022. Journal: Comput Intell Neurosci.

### 2.4. Data Transformation

After preprocessing, data transformation is done which is the initial stage of analysis. Data can be transformed in various ways, depending on the analysis procedure. In data transformation, the data are converted from one format to another format which may be more suitable for analysis. The new format can be a new destination system. The fMRI data are a 4-D data set that can be transformed into a 1-D data vector or can analyze as 2-D data with a different number of slices against the time.

### 2.5. Data Selection

The next step is data selection which has a convincing role in analysis, as it helps in extracting most of the significant information from the brain. The brain's slight behavior is changed during the task so data selection is necessary as most of the fMRI data slices do not have any contrast information. The size of fMRI data is large and less significant, so data selection becomes important in fMRI data. In the literature, various algorithms and methods are used for data selection like *t*-test, analysis of variance (ANOVA), entropy, Bhattacharyya distance, and others. In this study, *β* values found using *t* stats are used as initial features which are later refined using cumulants.

### 2.6. Feature Extraction

Feature extraction is an important part in which significant features should be extracted to make the analysis more valuable and reliable with improved accuracy. In fMRI data analysis, various features are already used such as region of interest, temporal-based feature selection, Dynamic causal modeling, features found using convolutional neural network, and many others. This essential part mostly uses statistical and mathematical methods to correlate different brain areas and helps in finding differences between the tasks. In the current study, various order cumulants are used as features that are given to the classifier for prediction.

### 2.7. Prediction

In this final step, prediction algorithms are used which help in determining the right classes for the testing data. Various algorithms and machine learning methods are used for this specific purpose such as support vector machine (SVM), linear discriminant analysis (LDA), Softmax, and others. The outcome of optimal predictor is in the form of accuracy based on true positives and true negatives which is later compared with various existing methods for validation.

The article "A Cumulants-Based Human Brain Decoding" was published in 2022. Journal: Comput Intell Neurosci.

## 3. Statistical Methodology

The proposed methodology of the paper is described as follows.

### 3.1. General Linear Model

The *t*-stats were found using a *t*-test from the raw data used as features for further analysis. These *t*-stats are found using the general linear model (GLM). The general linear model (GLM) is similar to statistical analyses [58], but it is also completely ideal both for various contextual and multifaceted variables. GLM is suitable for carrying out all parametric statistical tests with a dependent variable, like some factory configuration ANOVA, and designs with a combination of multiple variables (covariance analysis, ANCOVA). GLM is a key instrument for fMRI data analysis since being introduced by Friston and colleagues into the neuroimaging community [59] thanks to its versatility to integrate numerous, quantitative, and qualitative independent variables. In terms of a linear combination of the explanatory variables and an error term, a general linear model describes the response variable *Y*_*j*_.

(1) $$\begin{array}{c} Y_{j}=x_{j1}\beta_{1}+x_{j2}\beta_{2}+\cdots +x_{jL}\beta_{L}+\epsilon_{j}. \end{array}$$

The *β* parameters here are undisclosed to be estimated. *x*_*jL*_ is the explanatory variable, and *ϵ* is the error term that is arbitrary, with zero mean and variance *σ*. They are distributed independently and equally normally (i i d). The *xj* must be calculated *j*=1,2,…, *j* and *L*=1,2,…, *L* for each observation. In a single session, there are 400-time points mean value of *J* = 400, and 9 or 12 columns mean value of *L* = 9 or 12, according to the experiment performed. GLM can be written in matrix form which helps in deriving least squares parameter estimation. Equation (1) can be expanded as follows:

(2) $$\begin{array}{c} y_{1}=x_{11}\beta_{1}+x_{12}\beta_{2}+\cdots +x_{1L}\beta_{L}+\epsilon_{1},\\ ≔=≔,\\ y_{j}=x_{j1}\beta_{1}+x_{j2}\beta_{2}+\cdots +x_{jL}\beta_{L}+\epsilon_{j},\\ ≔=≔,\\ y_{J}=x_{J1}\beta_{1}+x_{J2}\beta_{2}+\cdots +x_{JL}\beta_{L}+\epsilon_{J}, \end{array}$$

where *Y* is the observing column vector *Y*=*y*_*j*_ *j*=1,2,…, *J*, *ϵ* is the error terms column vector, and *β* is the parameter column vector; *X* is the matrix of order *J* × *L*, and it is defined as the design matrix. The architecture matrix has one column or explaining element and one row per observation per model parameter.

### 3.2. Cumulants

The estimated parameters of GLM are fed to the optimal detector block as input data, which includes feature extraction and prediction stages after it has been transformed and selected. The extraction block calculates statistics called cumulative characteristics consisting of moments. Let *M*_*pq*_ represents the moments of input data *x*(*n*) which are estimated parameters of GLM and is calculated using

(3) $$\begin{array}{c} M_{pq}=E\left\{x{\left(n\right)}^{p-q}x^{*}{\left(n\right)}^{q}\right\}, \end{array}$$

where *E*{·} is defined as the expected value function which calculates the expected value of a random variable, and *p* and *q* are the indexed power term to define cumulants.

(4) $$\begin{array}{c} E\left\{x\right\}=\int_{-\infty }^{\infty }xf\left(x\right)dx\;. \end{array}$$

For the defined input data *x*(*n*), cumulants Ψ_*ij*_ of the second and fourth order are as follows [34]:

(5) $$\begin{array}{c} \Psi_{20}=E\left\{x^{2}\left(n\right)\right\},\\ \Psi_{21}=E\left\{{\left|x\left(n\right)\right|}^{2}\right\},\\ \Psi_{40}=M_{40}-3M_{20}^{2},\\ \Psi_{41}=M_{40}-3M_{20}M_{21},\\ \Psi_{42}=M_{42}-{\left|M_{20}\right|}^{2}-2M_{21}. \end{array}$$

The article "A Cumulants-Based Human Brain Decoding" was published in 2022. Journal: Comput Intell Neurosci.

### 3.3. Likelihood Ratio Test

The likelihood ratio test (LRT) is a test that is based on statistical analysis. It is a hypothesis test that tells how rightly two models can fit. This helps in choosing the best model between them [52]. The best model is chosen based on the likelihood function, means which maximizes the likelihood function.

Let *Y*=[*y*_1_, *y*_2_, *y*_3_,…, *y*_*k*_] represents the match scores for *K* individual matchers. The random variable *y*_*k*_ represents the kth matcher's match score, where *k*=1,2,…, *K*. Let's call the two classes *M*_0_ and *M*_1_, where *M*_1_ denotes a true positive (genuine) class and *M*_0_ denotes a true negative class. The conditional joint densities of the *k* match scores assigned to the first and second classes, respectively, are *p*(*Y|H*_0_) and *p*(*Y|H*_1_), where *Y*=[*y*_1_, *y*_2_, *y*_3_,…, *y*_*k*_], and assume that the null hypothesis is *H*_0_ and the alternative hypothesis is *H*_1_. Suppose the aim is to categorise the observed match score vector *Y* into one of two classes: *M*_0_ or *M*_1_. The null hypothesis should be dismissed, and the alternative hypothesis should be accepted. The likelihood ratio between null and alternative hypotheses is evaluated and analyzed for a decision threshold *θ*. The likelihood ratio test (LRT) is described as

(6) $$\begin{array}{c} LR\left(Y,H_{0},H_{1}\right)=\frac{p\left(Y|H_{0}\right)}{p\left(Y|H_{1}\right)}, \end{array}$$

where *Y* is the observed parameter, *p*(*Y|H*_0_) is the likelihood function for the null hypothesis which is evaluated for *Y*, similarly *p*(*Y|H*_1_) is the likelihood function for alternate hypothesis, and *θ* is the decision threshold which decides the acceptance or rejection of the null hypothesis. For example, if LR(*Y*, *H*_0_, *H*_1_) ≥ *θ*, the null hypothesis is accepted; otherwise, the alternative hypothesis is accepted.

The article "A Cumulants-Based Human Brain Decoding" was published in 2022. Journal: Comput Intell Neurosci.

In this study, Kernel density estimation (KDE) [53, 60]is used along with LRT for the acceptance or rejection of the null/alternative hypothesis. The approximation of probability density functions (pdfs) for training data is done using KDE. This is a nonparametric approach and has benefited because there is no permanent structure in KDE. Moreover, during estimation in KDE, all the data points are included in the analysis.

### 3.4. Proposed Algorithm

The collected data are first transformed into a simple matrix having rows and columns. This transformation is done using GLM based on *T*-values which is explained in the next section. The /beta values found using the design matrix are used as initial features and are comprehensively discussed in the performance evaluation section. SPM is used for the initial analysis of the data.

The kernel density function which is also known as kernel density estimation (KDE) is used for estimated class value; that is, the best match of each class with the test vector is found. Features from 50 to 5000 have been used and transformed these features using cumulants to reduce the size of the features vector. As a result, a maximum of eight features has been formed instead of 50 or 5000. Now, it is easy for kernel density function in terms of computation to process and find the best match during the fusion of match scores. Moreover, in this study, one-to-one results are extended to multiclass classification or multiclass decoding. In this case, one out of five classes was found using the proposed method. The detail is discussed in the result section. For cross-validation, Monte Carlo sampling is used, and the accuracy is found based on the average of 100 trials for each class to make the result reliable. The pseudo-code of the proposed methodology is depicted in Algorithm 1.

## 4. Results and Discussion

In this section, a detailed performance evaluation of the proposed optimal predictor is presented. In the experiment design, we had different images which were divided into five different categories. These images were taken from [61], and the categories were also made based on the same study. The images of five different classes are human, animal images, images of the building, images of natural scenes, and images of fruits. The design matrix is a matrix of values that consists of explanatory variables of different conditions or categories. Since there are five different categories, one variable (regressor) is defined for every category in the design matrix. A total of five variables are defined in the design matrix for five different conditions, and furthermore, for baseline and realignment parameters, separate variables (regressors) are used in the design matrix. Six realignment parameters are used to remove noise also known as nuisance regressors. There are five conditions, six nuisance regressors and a baseline, so a total of 12 regressors are used in the design matrix. The activity difference is found between the condition and the baseline for each category separately. For example, the activity difference between humans and baseline is shown in Figure 2. The statistical analysis of the image (Figure 2) is mentioned in the corresponding Table 1. Table 1 explains the degree of freedom, full width at half maximum (FWHM), voxel size, the position of voxels, *z*-values, number of clusters, number of significant voxels in each cluster, and other information. In the figure, the red arrow (<) shows the current location of the voxel (mostly the highest significant voxel), and the detail of this voxel is present in the first row (if highly significant) of Algorithm 1 with MNI coordinates, as also shown in red color. Since the significant voxels are important during analysis, so in the tables, the arrangement of voxels/clusters is shown in descending order means voxels/clusters with higher *T*-values are mentioned first. In Algorithm 1, the first three rows show the three most significant voxels of the most significant cluster while the first row shows the most significant voxels of the whole brain region for this task. In Figure 2, the brain activations are shown between humans and baseline while the behavior of the brain is the same for other sessions and participants. In the glass brain, it is observed that the activation area is the same for all the conditions (occipital region), but small differences can be seen among different categories. Generally, in the brain, there is always a small difference during the task concerning baseline [57], so further statistical analysis is required to find that difference. In the first-level analysis, those significant voxels are found which shows the activity differences during the condition to baseline for all sessions of every participant. These voxels are just the *β*-value for each trial and each voxel which was then used as a feature [17] for further analysis. In the existing study [17], these *β*-values are directly used as features and given to the classifier, that is, SVM to find the accuracy. On the other hand, in the current study, these features are further refined using a different order of cumulants, and finally, instead of using SVM, a different statistical technique is used, that is, LRT. SVM is the most common, reliable, and widely used classifier in neuroscience studies, but we propose different classification technique which shows better results compared to SVM.

The article "A Cumulants-Based Human Brain Decoding" was published in 2022. Journal: Comput Intell Neurosci.

During the analysis, the raw fMRI data were cleaned and passed through GLM to find the *β*-values which were used as initial features since fMRI data have a lot of features so feature reduction or refinement is very common. These initial features were refined and passed through LRT to predict the right class. The accuracy between 5 different classes was found using the one-to-one decoding method [62] between every two classes separately. The same procedure was repeated for other existing methods as shown in Table 2 to see the performance of the proposed method. There were a total of 10 one-to-one decoding combinations due to five different classes. The data were randomly distributed between 90% of training data and 10% of test data using Monte Carlo cross-validation. The 10% test data evaluate the performance of the proposed method. One-vs-one decoding results are shown in Figure 3 for all 10 combinations along with the number of features. In Figure 3, it is mentioned that the best results exist between 400 − 500 features in most of the cases. Classification accuracy is found for every individual participant but after combining the voxels of all three sessions. Classification is done one-against-one with multiclass SVM between every condition and participant separately. An uncorrected *p*-value of 0.001 is used to find the significance of every category.

It is very common in existing studies to take initial features from fMRI data (either raw data or *β*-value) and used SVM to find the prediction accuracy [17, 19, 63, 64]. In this study, we have proposed a different method that is more refined in terms of significant features and predictors. That's why to check the performance of the proposed system, the results are compared with various existing methods. The performance is checked based on accuracy and time which is one of the important factors. The proposed method is compared with various other methods mentioned in Table 2 and is also shown graphically in Figure 4. In linear discriminant analysis (LDA), *β*-values were taken as features as directly given to the classifier [17]. The features were not refined like the proposed method. Similarly, for the LibSVM case, same *β*-values were taken as features, and LibSVM was used as a classifier [65]. In the case of LRBSF, same features were used for the further process, but instead of any existing classifier, LRT was performed to find the best match of the predictor. In the existing study, LRT is used with refined features, that is, features found using cumulants.

The article "A Cumulants-Based Human Brain Decoding" was published in 2022. Journal: Comput Intell Neurosci.

For multiclass discrimination, the above-mentioned method (2 class likelihood ratio test) is extended to multiclass. Instead of choosing the best score match between two classes, we have chosen the match score with the highest value between the match score of the test vector and the class type. The result of multiclass decoding is shown in Figure 5 which indicates the accuracy against the number of features for all five classes simultaneously. The result is approximately 35% which is quite good as the chance in multidecoding is quite low, especially in 5 classes. Multiclass likelihood test is also used using LRBSF.

A comprehensive analysis of brain response and behavior is done, and the new features are used to improve the accuracy and response time. This study will help in various ways as it is contributing in many ways. The likelihood ratio test (LRT) is applied with cumulant features along with MVPA, and moreover, different classifiers are used to compare the results with LRT. This study gives the basic knowledge as well as focuses on advanced statistical and mathematical methods like LRT and the role of different levels of cumulants for the fMRI data set.

In short, this study is an addition to the existing methods proposed for fMRI data analysis. Since hardware limitations are not easy to overcome, new statistical and mathematical methods are always helpful in the analysis of neuronal data including fMRI, EEG, and MEG data.

## 5. Conclusion

In this study, a hybrid method is proposed which is an extension of various existing methods such as basic *β*-values or raw fMRI data are used as features for further analysis in most of the existing studies [17, 64]. In this study, these *β*-values are further polished to make the features more significant. Similarly, instead of using SVM which is the most common and widely technique of classification, a different statistical technique is used in neuroscience, that is, LRBSF. This technique is widely used in other applications [52, 66, 67] but has never been used in the analysis of fMRI data before. This LRBSF technique was initially introduced for fMRI data in 2017 by our research group [53]. In other words, this study is an extension and improvement of the previous study in terms of accuracy and response time. In the previous study, the response time was quite high which is improved in this study along with the accuracy. In short, this study includes numerous statistical and mathematical methods during the extraction of features. These new features are combined with the existing method, that is, LRBSF, which provides a novel hybrid method for the analysis of brain data acquired using fMRI. The new features which are introduced in the proposed algorithm are different levels of cumulants, and these features improved the overall accuracy from 66% to 70% while less response time is used than the previous one [53].

The article "A Cumulants-Based Human Brain Decoding" was published in 2022. Journal: Comput Intell Neurosci.

In the future, this algorithm can be applied to other modalities such as EEG and MEG. Moreover, other statistical methods such as the Gaussian mixture model and sequential Markov chain methods [27] and further levels of cumulants can be used with the existing methods to see the effect of additional features. This will be a new challenge for the researchers to work on various statistical techniques along with different modalities. The purpose is to achieve sufficient accuracy so that the neuroscience applications can widely be used especially BCI applications which can easily work with EEG data. By achieving acceptable accuracy, the fear among people can be reduced and actively build public support for neuroscience research. The goals should be set so that the public can recognize this field and share.

## Figures and Tables

**Figure 1:** System model for the analysis of fMRI data.

**Figure 2:** (a) (First-level analysis event-related design: human images vs baseline). (b) Design matrix which has 12 columns. In the design matrix, a number of variables are given horizontally, and trials are given vertically.

**Figure 3:** Average prediction accuracy of various combinations against the number of features. One-versus-one prediction for five different conditions which made 10 different combinations.

**Figure 4:** Comparison of various methods with the proposed method.

**Figure 5:** Multiclass decoding accuracy of five different classes. The chance level for five different classes is 20% while the best result is 35% according to the proposed method.

**Algorithm 1:** Optimal prediction algorithm.

**Table 1:** Static table for human vs baseline shows the degree of freedom, FWHM, voxel size, the position of voxels, *t*-value, cluster, and other details.

Statistics: p-value adjusted for search volume													
Set level		Cluster level				Peak level					mm	mm	mm
*p*	*c*	*p*_FEW_corr__	*q*_FDR_corr__	*k*_*E*_	*p*_uncorr_	*p*_FEW_corr__	*q*_FDR_corr__	*T*	*Z*	*p*_uncorr_			
0.002	45	0.000	0.000	2094	0.000	0.000	0.000	9.75	Inf	0.000	−15	−85	4
						0.000	0.000	9.67	Inf	0.000	−9	−91	l
						0.000	0.000	8.94	Inf	0.000	−27	−61	−2
		0.000	0.000	80	0.000	0.007	0.003	5.25	5.15	0.000	57	23	52
						0.328	0.047	4. 44	4 .38	0.000	54	32	34
		0.000	0.000	118	0.000	0.013	0.006	5.12	5.03	0.000	−45	−1	40
						0.029	0.010	4 .96	4 .88	0.000	−36	−4	61
						0.953	0.190	3.90	3.86	0.000	−45	−7	55
		0.005	0.001	39	0.000	0.026	0.010	4.98	4.9	0.000	24	−67	61
						l.000	0.676	3.35	3.32	0.000	30	−73	73
		0.004	0.001	40	0.000	0.037	0.012	4.91	4.83	0.000	−15	68	40
		0.000	0.000	248	0.000	0.071	0.020	4.77	4.70	0.000	27	11	70
						0.143	0.029	4.62	4.56	0.000	21	23	67
						0.221	0.037	4.52	4.46	0.000	9	17	73
		0.000	0.000	64	0.000	0.082	0.021	4.74	4.67	0.000	−24	−10	76
						0.628	0.081	4.24	4.19	0.000	−12	−19	85
						0.677	0.088	4.20	4.15	0.000	−18	−16	76
		0.205	0.021	16	0.008	0.082	0.021	4.74	4.67	0.000	75	−19	7
						l.000	0.777	3.27	3.25	0.001	69	−13	7
		0.000	0.000	123	0.000	0.087	0.021	4.73	4.66	0.000	33	47	1
						0.174	0.031	4.58	4.51	0.000	24	38	−11

Table shows three local maxima more than 0.8 mm apart. Height threshold: *T* = 3.11, *p* = 0.001 (1.000). Extent thresMd: *k*: 0 voxels. Expected voxels per cluster, <*k*> 2.012. Expected number of clusters, <*c* ≥ 28.41. FWEp: 4.846, FDRp: 4.427, FWEc: 27, FDRc: 14. Degree of freedom = [1.0, 3.91, 0]. FWHM: 7.7, 7.9, 7.6 mm mm mm; 2.6, 2.6, 2.5 (voxels}. Volume: 1481436 = 54868 voxels = 2846.7 resels. Voxel size: 3.0 3.0 3.0 mm mm mm; (resel: 17.29 voxels).

The article "A Cumulants-Based Human Brain Decoding" was published in 2022. Journal: Comput Intell Neurosci.

**Table 2:** Accuracy comparison of various methods using the fMRI data set.

Condition	LDA (%)	Deep learning (%)	Lib SVM (%)	LRBSF (%)	Proposed method (%)
Human vs animal	58.10	60.60	59.50	61.15	66.98
Human vs building	62.40	64.14	63.27	64.92	70.43
Human vs natural scenes	65.95	67.94	67.60	68.37	71.84
Human vs fruit	62.84	67.20	64.13	67.79	69.96
Animal vs building	65.25	68.80	66.23	69.42	71.71
Animal vs natural scenes	68.84	70.95	67.49	71.30	73.66
Animal vs fruit	66.12	67.17	67.74	67.73	68.88
Building vs natural scenes	58.54	60.10	57.68	59.47	67.72
Building vs fruit	62.29	64.25	63.93	64.62	70.10
Natural scenes vs fruit	62.47	64.84	63.92	65.52	69.82
Average	63.25	65.60	64.10	66.10	70.11

## Data Availability

The data were collected at the Hospital Universiti Sains Malaysia (HUSM). The details of the data are given in the manuscript. The processed data can be provided on demand. In our study, we have normal subjects, not patients, and we only examine the effect (for example, provider knowledge or attitudes). Therefore, the International Committee of Medical Journal Editors (ICMJE) on trial registrations is not required.
